The article "JQ1 suppresses tumor growth via PTEN/PI3K/AKT pathway in endometrial cancer" was retracted in 2026. Reasons: fabricated or falsified images; an official misconduct investigation; duplicated images; overlap with earlier publications.

# JQ1 suppresses tumor growth via PTEN/PI3K/AKT pathway in endometrial cancer

**DOI:** 10.18632/oncotarget.11631

**Published:** 2016-08-26

**Authors:** Haifeng Qiu, Jing Li, Leslie H. Clark, Amanda L. Jackson, Lu Zhang, Hui Guo, Joshua E. Kilgore, Paola A. Gehrig, Chunxiao Zhou, Victoria L. Bae-Jump

**Affiliations:** ^1^ Department of Obstetrics and Gynecology, the First Affiliated Hospital of Zhengzhou University, Zhengzhou, China; ^2^ Division of Gynecological Oncology, University of North Carolina at Chapel Hill, Chapel Hill, NC, USA; ^3^ Department of Oncology, the First Affiliated Hospital of Zhengzhou University, Zhengzhou, China; ^4^ Department of Gynecologic Oncology, Shandong Cancer Hospital and Institute, Jinan, China; ^5^ Lineberger Cancer Center, University of North Carolina at Chapel Hill, Chapel Hill, NC, USA

**Keywords:** endometrial cancer, JQ1, BRD4 inhibitor, PTEN/PI3K/AKT signal pathway, intrinsic resistance

## Abstract

Overexpression of c-Myc is associated with worse outcomes in endometrial cancer, indicating that c-Myc may be a promising target for endometrial cancer therapy. A novel small molecule, JQ1, has been shown to block BRD4 resulting in inhibition of c-Myc expression and tumor growth. Thus, we investigated whether JQ1 can inhibit endometrial cancer growth in cell culture and xenograft models. In PTEN-positive endometrial cancer cells, JQ1 significantly suppressed cell proliferation via induction of G1 phase arrest and apoptosis in a dose-dependent manner, accompanied by a sharp decline in cyclin D1 and CDK4 protein expression. However, PTEN-negative endometrial cancer cells exhibited intrinsic resistance to JQ1, despite significant c-Myc inhibition. Moreover, we found that PTEN and its downstream PI3K/AKT signaling targets were modulated by JQ1, as evidenced by microarray analysis. Silencing of PTEN in PTEN-positive endometrial cancer cells resulted in resistance to JQ1, while upregulation of PTEN in PTEN-negative endometrial cancer cells increased sensitivity to JQ1. In xenografts models of PTEN-positive and PTEN-knock-in endometrial cancer, JQ1 significantly upregulated the expression of PTEN, blocked the PI3K/AKT signaling pathway and suppressed tumor growth. These effects were attenuated in PTEN-negative and PTEN-knockdown xenograft models. Thus, JQ1 resistance appears to be highly associated with the status of PTEN expression in endometrial cancer. Our findings suggest that targeting BRD4 using JQ1 might serve as a novel therapeutic strategy in PTEN-positive endometrial cancers.

## INTRODUCTION

Endometrial cancer is one of the most common gynecological malignancies worldwide [1]. In the United States, both the incidence and mortality from endometrial cancer continues to rise, with an estimated 60050 new cases and 10470 deaths predicted in 2016 [2]. Obesity, diabetes and unopposed estrogen are well known risk factors for the development of endometrial cancer [3, 4]. Though outcomes in early-stage endometrial cancer are promising, the management of advanced stage and recurrent endometrial cancer remains challenging. Novel adjuvant therapies are needed for this subset of endometrial cancer [5].

c-Myc is a member of the Primary Response Genes (PRGs) that responds to the activation of Polymerase II [6]. c-Myc targets genes are responsible for encoding translational factors, nucleolar assembly components and ribosomal proteins integral to extracellular and intracellular signaling for cell growth, tissue regeneration and remodeling. In normal cells and cancer cells, c-Myc has been shown to manipulate cell proliferation, differentiation, apoptosis, cell cycle progression, adhesion, migration, angiogenesis and even metabolism through control on the transcription of its target genes [6–9]. Ectopic c-Myc expression in normal cells, particularly lymphocytes, results in the activation of checkpoints, such as p53, Arf or BimL, which cause apoptosis and/or cell cycle arrest [6]. Furthermore, enforced c-Myc expression in transgenic mice frequently results in hyperproliferation associated with reduced apoptosis in the target tissue [8, 10]. Knockdown of c-Myc in cancer cells *in vitro* uniformly reduces cell proliferation and in some instances, induces apoptosis and cell cycle arrest. In c-Myc transgenic mouse models, blocking ectopic c-Myc expression inhibits the growth of established tumors, suggesting that it is involved in tumor maintenance [11, 12].

The article "JQ1 suppresses tumor growth via PTEN/PI3K/AKT pathway in endometrial cancer" was retracted in 2026. Reasons: fabricated or falsified images; an official misconduct investigation; duplicated images; overlap with earlier publications.

There is accruing evidence that aberrant activity of c-Myc occurs in approximately 30% of human cancers, which results in enhanced tumor initiation and progression and correlates with advanced stage cancers, poor cellular differentiation, local and distant metastases and poorer prognosis [10, 13]. Overexpression of c-Myc is observed in 30–50% of patients with endometrial cancer and is associated with advanced stage, higher grade, distant metastasis and worse prognosis [14, 15]. Overexpression of c-Myc has been shown to cause increased cell proliferation, cell cycle progression and inhibition of apoptosis in endometrial cancer [16]. Moreover, endometrial cells transfected with c-Myc demonstrate altered morphology, focus formation, anchorage-independent growth, chromosomal alterations and increased tumor formation in athymic mice[17]. A recent study showed that SALL4, an epithelial-mesenchymal transition and drug resistance inducer, regulated cell invasion and drug resistance through the regulation of c-Myc in endometrial cancer [18]. This evidence suggests that c-Myc plays multiple roles in the pathogenesis of endometrial cancer and may serve as a potential therapeutic target for this disease.

The article "JQ1 suppresses tumor growth via PTEN/PI3K/AKT pathway in endometrial cancer" was retracted in 2026. Reasons: fabricated or falsified images; an official misconduct investigation; duplicated images; overlap with earlier publications.

There are currently several strategies for targeting c-Myc, including direct silencing of c-Myc by short interfere RNA (siRNA), inhibiting the key downstream genes of c-Myc and interrupting the dimerization between c-Myc and Max [10, 19]. Unfortunately, most of these approaches continue to be hampered by technical difficulties, pertaining largely to drug delivery and the fact that many c-Myc target genes are functionally redundant and/or cell type specific [20]. Recently, a small molecule, JQ1, was shown to be a potent c-Myc inhibitor. JQ1 was preliminarily designed as an inhibitor of bromodomain-containing proteins (BRDs), which could release BRDs from chromatin and abrogate their functions on regulating gene transcription [21]. Subsequent studies have shown that JQ1 effectively inhibits cell proliferation and tumor growth in a number of human malignancies, predominantly through inhibition of c-Myc and its downstream targets [22–24]. However, there is currently no evidence regarding the effect of JQ1 on cell growth in endometrial cancer *in vitro* or *in vivo*. In the present study, we investigated the effects of JQ1 on cell proliferation and tumor growth in endometrial cancer. We found that JQ1 significantly inhibited proliferation and tumor growth in endometrial cancer, with enhanced efficacy in PTEN-positive cell lines and xenografts.

## RESULTS

### JQ1 inhibited cell proliferation in Hec-1a and KLE cells

To investigate the effects of JQ1 on cell proliferation in endometrial cancer, we first employed the MTT assay to identify the cytotoxicity of JQ1 and measure the IC50 for each of the six endometrial cancer cell lines of interest. Cells were treated with JQ1 at varying concentrations for 72 hours. The MTT assay demonstrated a dose-dependent decrease in cell viability following treatment with JQ1 (Figure 1A). The IC50 values were 75 nM, 530 nM, 1950 nM, >10000 nM, >10000 nM, and >10000 nM for Hec-1a, KLE, ECC-1, Ishikawa, AN3CA, and RL95-2, respectively, after 72 hours of JQ1 treatment. Hec-1a and KLE cells were much more sensitive to JQ1 treatment than the other four cell lines.

**Figure 1:** JQ1 inhibited cell proliferation in endometrial cancer cells Six endometrial cancer cell lines were cultured for 24 hours and then treated with JQ1 at indicated doses in 96 well plates for 72 hours. (**A**) Cell proliferation was assessed by MTT assay. (**B**) JQ1 (100 nM) notably suppressed the colon formation in Hec-1a and KLE cells (*p* = 0.009 and 0.021 respectively). (**C**) JQ1 induced significant G1 phase arrest in Hec-1a and KLE cells after 24 hours of treatment with JQ1 (ranged from 0 nM to 1000 nM, *p* = 0.015 and 0.032 respectively). (**D**) In a time-lapse course, microarray analysis showed that JQ1 (500 nM) notably downregulated the mRNA expression of c-Myc, cyclin D1 and CDK4 in Hec-1a cells. (**E**) Western blotting results indicated that JQ1 inhibited cyclin D, CDK2, CDK4, CDK6 and cyclin E expression in a dose dependent manner after 24 hours of treatment. (**F**) JQ1 induced Annexin V expression in Hec-1a and KLE cells after 24 hours of treatment.

The article "JQ1 suppresses tumor growth via PTEN/PI3K/AKT pathway in endometrial cancer" was retracted in 2026. Reasons: fabricated or falsified images; an official misconduct investigation; duplicated images; overlap with earlier publications.

Considering that *in vitro* colony formation assay, measuring clonogenicity, has been shown to be an excellent indicator of long-term tumor survival and a predictor of the long-term anti-tumor effects of drugs [25], we subsequently assessed whether JQ1 treatment affected clonogenicity of Hec-1a and KLE cells. We observed that clonogenicity of both cell lines were significantly reduced after exposure to JQ1 for two weeks (*p* = 0.009 and 0.021, respectively, Figure 1B). Together, these results demonstrate suppressive effects of JQ1 on cell proliferation in Hec-1a and KLE cells.

We previously reported that JQ1 effectively induced cell cycle arrest and apoptosis in a dose dependent manner in ovarian cancer cells [26]. We also sought to evaluate the effect of JQ1 treatment on cell cycle distribution and apoptosis in the two JQ1 sensitive endometrial cancer cell lines (Hec-1a and KLE). Following 24 hours of treatment with JQ1, we found marked increase in G1 phase and reduced S phase in a dose-dependent manner in both Hec-1a and KLE cells compared to controls (*p* = 0.015 and 0.032, respectively, Figure 1C). To further investigate the mechanisms of JQ1 on cell cycle, we performed a time-lapse microarray analysis in Hec-1a cells after treatment of 100 nM JQ1 at varying time points (0 hour, 6 hours, 12 hours and 24 hours). We found that JQ1 inhibited RNA expression of c-Myc and cell cycle checkpoint related genes (Figure 1D). Western blotting was performed to confirm these findings and showed that JQ1 significantly inhibited protein expression of cell cycle checkpoints and c-Myc expression in Hec-1a and KLE cells after treatment JQ1 with 100 nM or higher doses (Figure 1E).

In order to determine whether the reduction of cell viability was related to apoptosis, we next detected apoptotic cells by using the Annexin-V and PI double staining assay on Cellometer. As shown in Figure 1F, the percentage of Hec-1a and KLE cells undergoing apoptosis significantly increased in a dose-dependent manner after 24 hours of treatment with JQ1 when compared to control. Hec-1a cells treated with 100 nM JQ1 were found to have increased the apoptotic rate more than two-fold compared to control (*p* = 0.021). KLE cells also underwent increased apoptosis at a JQ1 dose of 500 nM (*p* = 0.009). Collectively, our results suggested that JQ1 inhibited cell proliferation through induction of G1 phase cell cycle arrest and apoptosis in sensitive endometrial cancer cell lines.

The article "JQ1 suppresses tumor growth via PTEN/PI3K/AKT pathway in endometrial cancer" was retracted in 2026. Reasons: fabricated or falsified images; an official misconduct investigation; duplicated images; overlap with earlier publications.

### JQ1 inhibited the tumor growth in xenografts

In order to further evaluate the anti-tumor activity of JQ1 *in vivo*, we established a nude mouse model bearing Hec-1a cells. Ten days following injection of Hec-1a cells into the nude mice, the mice were treated with JQ1 (50 mg/kg/day, intraperitoneal injection) or placebo for 28 days. Tumor growth during treatment was monitored using calipers every four days. As shown in Figure 2A and 2B, JQ1 significantly suppressed tumor growth and reduced tumor weight in Hec-1a xenografts compared to control mice after 4 weeks of treatment (*p* < 0.001). In addition, JQ1 was shown to inhibit the expression of Ki-67, c-Myc and cyclin D1 in tumor tissues by immunohistochemical staining (IHC) (Figure 2C and 2D). These results indicate that JQ1 inhibits endometrial tumor growth *in vivo* via inhibition of expression of c-Myc and induction of cell cycle arrest.

**Figure 2:** JQ1 suppressed tumor growth in Hec-1a xenografts in nude mice JQ1 (intraperitoneal, 50 mg/kg/d, 5 days/week × 4 weeks) notably decreased tumor volume (**A**) and tumor weight (**B**) of Hec-1a xenografts in nude mice (*p* < 0.001). IHC results showed that JQ1 downregulated the protein expression of Ki-67, c-Myc and cyclin D1 in the Hec-1a xenografts (*p* = 0.039, 0.01 and 0.027, respectively) (**C** and **D**).

### JQ1 inhibited PI3K/AKT/S6 pathway via upregulating PTEN

Given that PTEN loss is the most common genetic abnormality in type I endometrial cancer, we investigate if PTEN status was related to the sensitivity to JQ1 in endometrial cancer cells. PTEN status was detected by western blotting in all six endometrial cancer cell lines. The results revealed that PTEN was abundant in the two JQ1 sensitive cell lines while extremely low in other cell lines (Figure 3A). We hypothesized that JQ1 may affect the expression of PTEN in these two sensitive cell lines. Microarray analysis was performed to test this hypothesis. Our microarray results found a dramatic increase in PTEN with a parallel decrease in its downstream targets (PI3K, AKT1/2/3, RPS6 and 4EBP1) after treatment with JQ1 in the Hec-1a cells (Figure 3B). Confirmatory western blot assays showed that there was increased PTEN expression and decreased phosphorylation of AKT and S6 in both the Hec-1a and KLE cells, following 24 hours of JQ1 treatment (Figure 3C, 3D and Supplementary Figure S1). These findings suggest that the sensitivity to JQ1 is associated with PTEN function and the PI3K/AKT/S6 pathway in these endometrial cancer cell lines.

The article "JQ1 suppresses tumor growth via PTEN/PI3K/AKT pathway in endometrial cancer" was retracted in 2026. Reasons: fabricated or falsified images; an official misconduct investigation; duplicated images; overlap with earlier publications.

**Figure 3:** JQ1 increased the expression of PTEN and blocked the PI3K/AKT/S6 pathway (**A**) Western blotting results showed the status of PTEN expression in six endometrial cancer cell lines. (**B**) Microarray results indicated that JQ1 increased the mRNA of PTEN and inhibited the PI3K/AKT/S6 signals in Hec-1a cells. Q1 significantly increased the protein expression of PTEN and decreased phospho-AKT/phospho-S6 expression in Hec-1a (**C**) and KLE (**D**) cells after 24 hours of treatment.

### PTEN status affected cellular sensitive to JQ1 *in vitro*

To further investigate the underlying mechanisms of JQ1 inhibition of cell proliferation in PTEN-positive cells, we transfected the specific shRNA-PTEN plasmids into Hec-1a and KLE cells. This generated two cell lines with stable knockdown of PTEN and accompanying upregulation of phosphorylated-AKT (Figure 4A). Cell proliferation was then assessed by MTT assay. We hypothesized that the inhibition of PTEN protein expression would decrease the cellular sensitivity to JQ1 treatment. In support of our hypothesis, knockdown of the PTEN gene in the both cell lines induced significant cellular resistance to JQ1 (Figure 4B and 4C) and increased the IC50 for both cell lines (75 nM versus 420 nM for Hec-1a, 530 nM versus 3350 nM for KLE, *p* = 0.008 and 0.011, respectively). We next examined the effect of JQ1 on cell cycle disruption in PTEN knockdown cells. Similarly, the loss of PTEN in both cell lines resulted in loss of the previously identified G1 phase arrest induced by JQ1 at dose of 500 uM (*p* = 0.025 and 0.019, respectively, Figure 4D and 4E).

**Figure 4:** The sensitivity of JQ1 is dependent on the status of PTEN in endometrial cancer cells (**A**) Knockdown PTEN expression by a specific shRNA-PTEN significantly reduced the expression of PTEN in the two endometrial cancer cell lines (**B** and **C**) Hec-1a and KLE cells with PTEN loss became less sensitive to JQ1 (IC50 = 420 nM for Hec-1a and 3350 nM for KLE). (**D** and **E**) PTEN loss eliminated the G1 phase arrest caused by JQ1 in Hec-1a and KLE cells after 24 hours of treatment (*p* = 0.025 and *p* = 0.019 respectively). Figure D and E represent one of three independent experiments. (**F**) The protein level of PTEN was notably elevated in AN3CA and Ishikawa cell lines with stably transfection of pcDNA3-PTEN plasmids. (**G** and **H**) the AN3CA and Ishikawa cells transfected by pcDNA3-PTEN significantly increased the sensitivity of JQ1 compared to their parental cells after 72 hours of treatment (*p* = 0.006 and *p* = 0.013 respectively). (**I** and **J**) JQ1 induced significant G1 phase arrest in AN3CA and Ishikawa cells with PTEN overexpression after 24 hours of treatment (*p* = 0.012 and *p* = 0.02 respectively). Figure (I and J) represent one of three independent experiments.

The article "JQ1 suppresses tumor growth via PTEN/PI3K/AKT pathway in endometrial cancer" was retracted in 2026. Reasons: fabricated or falsified images; an official misconduct investigation; duplicated images; overlap with earlier publications.

To further address our hypothesis, PTEN-negative and JQ1 insensitive cell lines, AN3CA and Ishikawa, were transfected with wild-type PTEN. Cell lysates were analyzed by western blotting for PTEN expression. Transfection of PTEN increased wild-type PTEN expression levels with a sharp decrease in phosphorylation of AKT in AN3CA and Ishikawa cells (Figure 4F). MTT assay was then performed on the wild-type PTEN AN3CA and Ishikawa cell lines, and increased sensitivity to JQ1 treatment was noted compared to the parent AN3CA and Ishikawa cell lines (Figure 4G and 4H, IC50 = 4100 nM for AN3CA and 2600 nM for Ishikawa, respectively, *p* = 0.006 and 0.013, respectively). Similarly, cell cycle analysis showed that JQ1 increased G1 phase arrest in wild-type PTEN AN3CA and Ishikawa cell lines (Figures 4I and 4J, *p* = 0.012 and 0.02, respectively) as compared to the parent cell lines. Collectively, our results demonstrate that the anti-tumor activity of JQ1 in endometrial cancer depends on the PTEN functional status of the endometrial cancer cells.

### The anti-tumor activity of JQ1 depended on PTEN status *in vivo*

To better elucidate the correlation between PTEN status and tumor sensitivity to JQ1, we established four nude mice models (Balb b/c nude mice) using parental Hec-1a cells, Hec-1a cells with PTEN knockdown, parental AN3CA cells and AN3CA cells with PTEN knock-in. Beginning ten days after cell injection, the mice were treated with JQ1 at 50 mg/kg/day for four continuous weeks. The mice showed tolerance to JQ1 injections and maintained normal activities. Consistent with our results *in vitro*, Hec-1a xenografts with knockdown of PTEN showed less response to four weeks of JQ1 treatment compared to their parental Hec-1a xenograft counterparts, resulting in increased tumor weight in the PTEN knockdown mice (Figure 5A and 5B). The analysis of immunostaining staining showed that an increase of the protein levels of Ki-67 and phosphorylated-AKT was observed in tumor tissues in Hec-1a xenografts with PTEN-knockdown (*p* = 0.05 and 0.003, respectively, Figure 5C and 5D). On the contrast, the AN3CA xenografts with PTEN knock-in became much more sensitive to JQ1 than their parental ones after 4 weeks of treatment, accompanied by a decrease in tumor weights (Figure 5E and 5F), while IHC results showed that expression levels of Ki-67 and phosphorylated-AKT were decreased in the tumor tissues in AN3CA xenografts with PTEN knock-in treated with JQ1 (*p* = 0.041 and 0.018, respectively, Figure 5G and 5H). These results confirm that JQ1 inhibition of endometrial tumor growth dependent is dependent on PTEN function *in vivo.*

The article "JQ1 suppresses tumor growth via PTEN/PI3K/AKT pathway in endometrial cancer" was retracted in 2026. Reasons: fabricated or falsified images; an official misconduct investigation; duplicated images; overlap with earlier publications.

**Figure 5:** Tumor sensitivity to JQ1 was dependent on PTEN status *in vivo* (**A**) The Hec-1a xenografts with PTEN loss presented resistance to JQ1 after 4 weeks of treatment (*p* = 0.039). (**B**) PTEN loss in Hec-1a xenografts significantly increased tumor weights (*p* = 0.027) (**C** and **D**) IHC results showed that the protein expression of Ki-67 and phospho-AKT were increased in Hec-1a xenografts with PTEN-knockdown (*p* = 0.05 and 0.003, respectively). (**E**) AN3CA xenografts with PTEN knock-in became much more sensitive to JQ1 than their parental ones after 4 weeks of treatment (*p* = 0.014). (**F**) The tumor weights were also decreased in AN3CA xenografts with PTEN loss (*p* = 0.036). (**G** and **H**) The expression of Ki 67 and p-AKT were decreased in the tumor tissues with abundant PTEN in AN3CA xenografts (*p* = 0.041 and 0.018, respectively).

### JQ1 inhibited cell proliferation in primary cultures of endometrial cancer

Previous studies have demonstrated that assessing the sensitivities of drugs in cancer cells in primary culture can provide clinically relevant information for the optimization of the cancer patient's treatment [25]. Therefore, we further investigated the effects of JQ1 on tumor cell growth in primary cultures of endometrial cancer patients using the MTT assay. Twenty-eight tissue samples were obtained from patients undergoing primary surgical staging for endometrial cancer. After 72 hours of treatment with JQ1, 17 of 28 individual patient cultures responded to treatment with significant growth inhibition at doses up to 10 μM. Ten of the 17 sensitive cultures exhibited significantly reduced cell proliferation under JQ1 treatment, with a range of IC50 values from 22 to 530 nM (Table 1). The cell cultures with positive PTEN expression were significantly more sensitive to JQ1 than the PTEN-negative cells (*p* < 0.001, Table 1, Figure 6A and Supplementary Figure S2), consistent with our previous findings in established endometrial cancer cell lines. In order to determine if the level of PTEN protein expression correlated with sensitivity to JQ1 in each primary culture case, we detected the expression of PTEN using western blotting in the 28 untreated primary cell cultures. The results revealed varying levels of PTEN expression in 11 primary culture samples and negative PTEN expression in the remaining 17 primary culture samples (Table 1, Figure 6B). Analyzing this data using a linear regression model, we find that PTEN-positive cultures responses to JQ1 were dependent upon the level of PTEN protein expression (R^2^ = 0.3806, *p* = 0.0432, Figure 6C). Moreover, we detected that JQ1 significantly arrested cell cycle at G1 phase and inhibited the expression of cyclin D1 and CDK4 in the PTEN-positive but not in PTEN-negative primary cultures (Figure 6D and 6E).

The article "JQ1 suppresses tumor growth via PTEN/PI3K/AKT pathway in endometrial cancer" was retracted in 2026. Reasons: fabricated or falsified images; an official misconduct investigation; duplicated images; overlap with earlier publications.

**Table 1:** Summary of patients' information for primary culture

Case No.	Stage	Grade	Histologic subtype	IC50(nM)	PTEN status
1	IA	1	Endometrioid	36	positive
2	IB	1	Endometrioid	320	positive
3	IA	1	Endometrioid	775	negative
4	IA	2	Endometrioid	22	positive
5	IB	1	Endometrioid	2600	negative
6	IA	2	Endometrioid	220	positive
7	IA	2	Endometrioid	190	positive
8	IA	1	Endometrioid	2260	negative
9	IA	2	Serous	> 10000	negative
10	IB	1	Endometrioid	> 10000	negative
11	IA	1	Endometrioid	78	positive
12	IB	1	Endometrioid	139	positive
13	II	1	Endometrioid	650	negative
14	IA	2	Endometrioid	> 10000	negative
15	IIIA	3	Endometrioid	3300	negative
16	IB	1	Endometrioid	615	positive
17	IA	1	Endometrioid	1850	negative
18	IA	1	Endometrioid	86	positive
19	IIIC1	2	Endometrioid	950	negative
20	IIIC1	3	Endometrioid	120	negative
21	IA	1	Endometrioid	830	positive
22	IIIC1	3	Endometrioid	835	negative
23	IIIA	1	Endometrioid	1850	negative
24	IIIC1	3	Undifferentiated	> 10000	negative
25	IA	1	Endometrioid	530	negative
26	IIIC1	2	Serous	1600	positive
27	IVB	3	Undifferentiated	500	negative
28	IIIC2	3	Undifferentiated	> 10000	negative

**Figure 6:** PTEN status related to the sensitivity to JQ1 in the primary cultures of endometrial cancer (**A**) The primary cultures with negative PTEN were insensitive to JQ1 compared with those with positive PTEN expression (*p* < 0.001). (**B**) Western blotting showed the status of PTEN expression in the primary cultures of endometrial cancer. (**C**) The sensitivity to JQ1 in PTEN-positive cultures was dependent upon the level of PTEN protein expression using a linear regression model (*R*^2^ = 0.3806, *p* = 0.0432). (**D** and **E**) JQ1 caused notably G1 phase arrest and decreased protein expression of cyclin D1 and CDK4 in Case 7 (PTEN-positive), but not in case 10 (PTEN-negative), after 24 hours of treatment.

## DISCUSSION

The key to successful targeted molecular therapies is the identification of key oncogenes whose effective inhibition can induce apoptosis, cell cycle arrest and/or cellular differentiation in cancer cells. Accumulating *in vitro* and *in vivo* evidence suggest that c-Myc is an excellent target for anti-cancer therapeutics due to its involvement in almost every step of tumor initiation and progression [10, 13]. Over the last few years, several small molecular inhibitors that specifically target c-Myc have been developed. Some of these inhibitors have demonstrated promise and will be investigated in upcoming clinical trials [19, 27, 28]. Of the c-Myc inhibitors, JQ1 has shown particular efficacy in inhibiting the expression of c-Myc and its downstream genes. Furthermore, in a large panel of human cancer cell lines, animal models and human primary tumor samples, JQ1 has been found to increase G1 cell cycle arrest and induce apoptosis and cellular senescence [21–24]. JQ1 has also been found to have synergistic effects on the inhibition of tumor cell proliferation when combined with fulvestrant, an estrogen receptor antagonist, in breast cancer [29], γ-secretase inhibitors in T cell acute lymphoblastic leukemia [30] and histone deacetylase inhibitors in murine lymphoma [31].

The article "JQ1 suppresses tumor growth via PTEN/PI3K/AKT pathway in endometrial cancer" was retracted in 2026. Reasons: fabricated or falsified images; an official misconduct investigation; duplicated images; overlap with earlier publications.

Given that amplification and/or overexpression of c-Myc is frequently detected in human endometrial cancer and correlates with worse overall prognosis [14], we investigated the inhibitory effects of JQ1 in endometrial cancer both *in vitro* and *in vivo*. Our results show that JQ1 significantly suppresses cellular proliferation and induces G1 phase cell cycle arrest in endometrial cancer cells that express PTEN through inhibition of c-Myc and cell cycle checkpoints in both PTEN-positive established cell lines and primary cultures of human endometrial cancer. Moreover, *in vivo*, JQ1 also significantly reduced tumor growth in PTEN-positive Hec-1a and PTEN knock-in AN3CA xenografts. Given the potent anti-cancer effects and mild toxicities seen in a large body of *in vitro* and pre-clinical studies, JQ1 may offer considerable promise in the treatment of PTEN-positive endometrial cancer, among others [12, 24, 32].

PTEN loss is the most common molecular alteration in endometrial cancer due to mutation, deletion and promoter hypermethylation [33]. PTEN mutations have been identified in up to 83% of endometrioid carcinomas and 55% of precancerous lesions [34]. PTEN protein has both lipid and protein phosphatase activity with each serving different functions including regulation of cell cycle, apoptosis, adhesion, invasion and inhibition of the PI3K/AKT pathway. Knock-out mice rendered heterozygous or homozygous for PTEN developed endometrial hyperplasia, atypical hyperplasia and endometrial carcinoma [35, 36]. Thus, loss of PTEN is likely an early event in endometrial tumorigenesis and likely initiated in response to known hormonal risk factors for endometrial cancer such as obesity and insulin resistance. The loss of PTEN or alterations of PTEN expression results in aberrant cell growth and apoptotic escape. PTEN restoration results in inhibition of cell proliferation, G1 phase cell cycle arrest, induction of apoptosis and inhibition of telomerase activity [37, 38]. The loss of PTEN has been implicated in cellular resistance to several oncoprotein targeting agents including imatinib, EGFR inhibitors, fulvestrant and BRAF inhibitors [39, 40]. A recent study reported that intrinsic resistance to JQ1 was found in non-small cell lung cancer with mutant KRAS and LKB1, while cells with only mutant-KRAS still were sensitive to JQ1 [41]. Our data finds that PTEN-positive cell lines are highly sensitive to JQ1 when compared to PTEN-negative cell lines. In addition, data from both microarray and western blotting support that JQ1's anti-tumorigenic effects are dependent on PTEN expression. These results suggest that PTEN status may serve as a crucial biomarker of intrinsic resistance to JQ1 and PTEN expression testing will be important in future trials evaluating JQ1 for cancer treatment [42].

The article "JQ1 suppresses tumor growth via PTEN/PI3K/AKT pathway in endometrial cancer" was retracted in 2026. Reasons: fabricated or falsified images; an official misconduct investigation; duplicated images; overlap with earlier publications.

PTEN is a dual-phosphatase that negatively regulates AKT activity. Loss of PTEN and activation of the PI3K/AKT pathway results in resistance to targeted therapies with small molecule compounds in some cancers including endometrial cancer, as discussed above. Down-regulation of PTEN in breast cancer cells results in trastuzumab-resistance both *in vitro* and *in vivo*, but the use of PI3K inhibitors, such as LY294002 and Wortmannin, rescues PTEN loss-induced trastuzumab resistance [43]. Data from clinical trials has demonstrated that breast patients with negative PTEN expression have significantly worse response to trastuzumab and shorter overall survival than those with positive PTEN expression, suggesting that PTEN status can be used as a predictive marker for trastuzumab treatment in breast cancer [43]. Recent studies also support that PTEN down-regulation can be used as a biomarker to predict low response to the EGFR inhibitors (cetuximab and gefitinib) in colorectal and lung cancer [44, 45]. In this study, we downregulated or upregulated the expression of PTEN in JQ1-sensitive or resistant cells by stable transfection, and found that knockdown of PTEN induced significant resistance to JQ1 and knock-in of PTEN re-sensitized the cells to JQ1 *in vitro* and *in vivo*. The effects of PTEN on JQ1-sensitivity are believed to be due to inhibition of the PI3K/AKT pathway. Activation of PI3K/AKT pathway has been shown to be responsible for loss of PTEN function induced drug resistance. Indeed, a panel of small molecular drugs targeting PI3K and mTOR pathway were proven to be more effective in patients with PTEN loss or PTEN mutation [46, 47]. However, a study in glioblastoma found that neither hyperactivated AKT nor p53/Rb loss has an effect on the cellular sensitivity to JQ1 [23], indicating that PTEN status as predictive marker may be associated with certain types of cancer (such as endometrial cancer) and not others.

The article "JQ1 suppresses tumor growth via PTEN/PI3K/AKT pathway in endometrial cancer" was retracted in 2026. Reasons: fabricated or falsified images; an official misconduct investigation; duplicated images; overlap with earlier publications.

Assessment of chemotherapeutic drug sensitivities using primary culture cancer cells provides clinically relevant information for the optimization of cancer treatment strategies [48]. In a panel of 28 primary cell cultures from endometrial cancer patients undergoing primary surgery, positive PTEN expression was correlated with JQ1 inhibition of cell growth and induction of cell cycle arrest. The level of PTEN protein expression in untreated cells from primary cultures was associated with sensitivity to JQ1. Further analysis found that c-Myc protein expression was not associated with sensitivity to JQ1 in these cells (data not shown). These results provide further support that inhibition of bromodomain and extra terminal proteins (BET) may be used as a potential therapeutic approach in endometrial cancer patients with PTEN expression. As for endometrial cancer patients with PTEN loss, combination therapy with PI3K inhibitors (to overcome the PTEN loss mediated resistance) for bromodomain inhibitors, including JQ1, should be explored.

In summary, targeting c-Myc via JQ1 was found to have promising anti-tumorigenic activity in PTEN-positive endometrial cancer cell lines, primary cultures and xenografts. Our work suggests a causal link between JQ1 treatment and the PTEN/PI3K/AKT pathway in endometrial cancer *in vitro* and *in vivo*. We believe our present study establishes a fundamental relationship of inhibition of c-Myc by JQ1 to cell proliferation, apoptosis and cell cycle arrest in endometrial cancer cells, providing a molecular basis for the use of bromodomain inhibitors for endometrial cancer treatment.

## MATERIALS AND METHODS

### Cancer cell lines and reagents

The cell lines used in this study were ECC-1, KLE, RL95-2, Ishikawa, AN3CA, and Hec-1a. For the ECC-1 cells, RPMI 1640 medium with 5% fetal bovine serum (FBS) was used. For the KLE and RL95-2 cells, DMEM/F12 with 10% FBS was used. For the Ishikawa and AN3CA cell s, MEM with 5% FBS was used. For the Hec-1a cells, McCoy's 5A with 10% FBS was used. All cells were purchased from ATCC (American type culture collection, USA) and cultured at 37°C in a humidified incubator containing 5% CO_2_. All the reagents used in this study were purchased from Sigma-Aldrich (St. Louis, MO), unless otherwise stated. JQ1 was kindly gifted by Dr. James E. Brander (Harvard Medical School, MA). All the primary antibodies for phosphorylated-S6, pan-S6, phosphorylated-AKT, pan-AKT, cyclin D1, CDK6, CDK4 and Ki-67 were obtained from Cell Signaling Technology (Danvers, MA, USA). Enhanced chemiluminescence (ECL) detection reagents were purchased from GE Health care (Piscataway, NJ).

The article "JQ1 suppresses tumor growth via PTEN/PI3K/AKT pathway in endometrial cancer" was retracted in 2026. Reasons: fabricated or falsified images; an official misconduct investigation; duplicated images; overlap with earlier publications.

### Western blotting

Total protein was extracted from tumor cells or tissues using RIPA buffer (Thermo Fisher, MA) and quantified by BCA assay (Thermo Fisher). Equal amounts of total protein (50 μg) were separated by 12% SDS-PAGE, transferred onto PVDF membrane, blocked in 5% non-fat milk for 1 hour and incubated with the primary antibodies (1:1000 diluted) overnight at 4°C. On the second day, the membrane was incubated with appropriate secondary antibodies for 2 hours at room temperature and then the specific bands were developed using ECL buffer. The results were quantified using the Alpha Innotech Imaging System (San Leandro, CA). β-actin (Sigma-Aldrich, 1:2000 diluted) was used as the endogenous control. The experiments were performed in triplicate and repeated at least three times.

### Tissue samples collection and primary cell culture

Twenty-eight consecutive pathologically diagnosed endometrial cancer samples were collected from UNC Hospital (Chapel Hill, NC, USA) and the First Affiliated Hospital of Zhengzhou University (Zhengzhou, China) from September 2012 to December 2014. All patients provided written consents and approval was obtained from the respective Institutional Review Board (IRB) committees. Tumors were staged and graded according to the criteria of the International Federation of Obstetrics and Gynecology (FIGO) 2009. All patient and corresponding tumor information is summarized in Table 1. For the primary culture, the fresh tumor tissues were immediately washed three times with Hank's Buffered Salt Solution (HBSS), gently minced using a scalpel, then placed in DMEM/F12 medium containing 10% FBS. These cells were digested in a mixture of 0.1% collagenase IA, 100 U/ml penicillin and streptomycin for 0.5 to 1 hour at 37°C. After centrifuging twice with PBS solution, cells were resuspended and diluted to 1 × 10^5^ cells/ml with DMEM/F12 medium. Next, 2 × 10^4^ cells/well were seeded into 96-well plates for MTT assay, and 3 × 10^5^ cells/well were plated in 6-well plates for cell cycle analysis. Cells were incubated overnight before treatment with JQ1. Cellular growth curves and cell cycle phase distribution were measured after 24 and 72 hours of JQ1 treatment, respectively.

### MTT assay

The effect of JQ1 on cellular growth was determined by MTT assay. Briefly, 4 × 10^3^ cells/well were seeded into 96-well plates and incubated overnight. Plates were then treated with JQ1 at different concentrations for 72 hours. Five μl of MTT solution (5 mg/ml) was added to each well and incubated for 1 hour. The formazan crystals were dissolved in 100 μl of DMSO. The absorbance was measured at 570 nm with a microplate reader (Tecan, Morrisville, NC). Each experiment was performed in triplicate to assess for consistency of results.

The article "JQ1 suppresses tumor growth via PTEN/PI3K/AKT pathway in endometrial cancer" was retracted in 2026. Reasons: fabricated or falsified images; an official misconduct investigation; duplicated images; overlap with earlier publications.

### Colony formation assay

One hundred cells/well were plated into 6-well plates and incubated overnight. The cells were then treated with 100 nM of JQ1 on the following day and further cultured at 37°C for two weeks. After two weeks, the cells were fixed using chilled 10% methanol for 10 minutes and then stained in 0.5% Gimsa solution for 15 minutes. The excess staining solution was gently rinsed and colonies containing more than 50 cells were counted using an optical microscope. Cells were also treated with DMSO as the negative control. Colony formation assays were performed in duplicate for consistency of results.

### Cell cycle analysis

Cell cycle distribution was measured by the PI staining method on Cellometer (Nexcelom, MA). Briefly, 1.5 × 10^5^ cells/well were seeded into 6-well plates and treated with JQ1 for 24 hours. Control cells were treated with DMSO. After treatment, cells were fixed in chilled 90% methanol and stored at -20°C for at least 2 hours. Next, the cells were washed with PBS and incubated with 50 μl RNase A solution. 50 μl of PI staining solution (containing 2 mg/ml PI, 0.1 mg/ml Azide, and 0.05% Triton X-100) was added to the cell suspension. The final mixture was incubated for 15 minutes in the dark before being analyzed using the Cellometer. Cell cycle analysis was performed by FCS Express 4 software (De Novo Software, Los Angeles, CA). All experiments were performed in triplicate to assess for consistency of response.

### Apoptosis assay

Apoptosis was detected using the PI/Annexin V staining kit (Thermo Fisher) on Cellometer. Briefly, 1.5 × 10^5^ cells/well were seeded into 6-well plates and incubated overnight. Cells were then treated with different doses of JQ1 for 24 hours. Control cells were treated with DMSO. The cells were harvested and stained by PI (2 mg/ml) and Annexin V (100 μg/ml, Biolegend, CA) for 15 minutes in the dark. The apoptotic cells were detected by Cellometer and the results were analyzed by the FCS Express 4 software. All experiments were performed in triplicate to assess for consistency of response.

### Establishment of the stably transfected cell lines

The pcDNA3-PTEN and shRNA-PTEN plasmids were obtained from Addgene (plasmid 10759 and 10669, Cambridge, MA). The pcDNA3-PTEN or shRNA-PTEN plasmids were transfected into AN3CA or Hec-1a cells using FuGENE HD following manufacturer instructions (Roche, Mannheim, Germany). Cells were then maintained with G418 (500 μg/ml, Gibco, CA) to select the stably transfected clones. The cells transfected with empty plasmids were set as the negative control. PTEN protein expression was determined using western blotting.

The article "JQ1 suppresses tumor growth via PTEN/PI3K/AKT pathway in endometrial cancer" was retracted in 2026. Reasons: fabricated or falsified images; an official misconduct investigation; duplicated images; overlap with earlier publications.

### Tumor xenografts growth assay

Six-week-old female mice with severe combined immunodeficiency were used for this assay. All mice were handled according to protocols approved by the ethics committee of Zhengzhou University. In brief, 1 × 10^6^ cells were injected subcutaneously into the right flank of mice. Ten days after injection, JQ1 (IP, 50 mg/kg/d) or DMSO was administered to different groups of mice. The tumor size was measured using calipers every four days. The tumor volume was calculated using the formula (length × width^2^)/2. All the mice were sacrificed after four weeks of JQ1 treatment and the tumor tissues were collected for further analysis.

To study the anti-tumor functions of JQ1, two groups of mice were used (*n* = 4 in each group): Hec-1a+DMSO and Hec-1a+JQ1. To confirm the effects of PTEN on JQ1 resistance, another four groups of mice were used (*n* = 4 in each group): Hec-1a+JQ1, Hec-1a-PTEN^loss^+JQ1, AN3CA+JQ1 and AN3CA-PTEN^gain^ +JQ1.

### Microarray analysis

Microarray studies were performed as previously described [49]. Briefly, 1.5 × 10^5^ Hec-1a cells/well were plated in 6-well plates and treated with JQ1 (500 nM) for 0, 6, 12 and 24 hours. Total RNA was extracted using the RNAeasy Kit (Qiagen, Hilden, Germany). Hybridization was performed using a UNC-customized microarray from Agilent Technologies (Santa Clara, CA). The results were analyzed with GenePix Pro 4.1 and uploaded onto the Microarray Database of UNC at Chapel Hill (https://genome.unc.edu/). These assay was performed in duplicate for consistency of results.

### Immunohistochemical staining (IHC)

Tumor tissues from mice were formalin-fixed and paraffin-embedded. After rehydration and antigen retrieval, the slides (thickness = 4 μm) were incubated with primary antibodies: anti-Ki-67 (1:300), anti-c-Myc (1:100), anti-cyclin D1 (1:50), anti-PTEN (1:100) and anti-p-AKT (1:50). The staining was visualized using DAB (Invitrogen, CA). The slides were scored by two pathologists.

### Statistical analysis

Results were compared by Student's *t* test and data were expressed as mean ± S.E. χ^2^ test was used for the analysis of 2 × 2 tables. Statistical significance was defined to be *p* < 0.05.

## SUPPLEMENTARY MATERIAL FIGURES


